The article "Application Value of Contrast-Enhanced Ultrasound Combined with Enhanced MR Scanning in Patients with Intrahepatic Cholangiocarcinoma" was retracted in 2023. Reasons: suspected computer-generated content; unreliable results or conclusions; concerns about the data; concerns about the results or conclusions.

# Application Value of Contrast-Enhanced Ultrasound Combined with Enhanced MR Scanning in Patients with Intrahepatic Cholangiocarcinoma

**DOI:** 10.1155/2022/6402646

**Published:** 2022-03-31

**Authors:** Mingming Zhang, Yan Liu, Lei Han, Guixiang Zhang

**Affiliations:** ^1^Department of Ultrasound, Ganyu District People's Hospital of Lianyungang City, Lianyungang 222100, China; ^2^Magnetic Resonance Room, Ganyu District People's Hospital of Lianyungang City, Lianyungang 222100, China; ^3^Department of Hepatobiliary Surgery, Ganyu District People's Hospital of Lianyungang City, Lianyungang 222100, China

## Abstract

**Objective:**

To explore the clinical application effect of contrast-enhanced ultrasound (CEUS) combined with enhanced MR scanning in patients with intrahepatic cholangiocarcinoma (ICC).

**Methods:**

90 patients with ICC admitted to Ganyu District People's Hospital of Lianyungang City from June 2017 to June 2018 were selected as the research objects and randomly divided into control group and experimental group, with 45 cases in each group. The control group was tested by CEUS, and the experimental group was tested by CEUS combined with enhanced MR scanning. The test results of the two groups were compared, and the benign and malignant indicators of the two groups were detected.

**Results:**

The rate of lesion detection, accuracy of localization qualitative accuracy, and diagnosis coincidence rate of the experimental group were significantly better than those of the control group (*p* < 0.05). The lesion length, tube wall thickness, and enhancement ratio of triple-phase multislice CT scan of the experimental group were lower than the control group (*p*＜0.05).

**Conclusions:**

CEUS combined with enhanced MR scanning has high sensitivity and specificity and can significantly improve the accuracy of the detection results. It provides scientific and accurate scientific basis for clinical treatment and diagnosis of ICC, which is worthy of popularization and application.

## 1. Introduction

Intrahepatic cholangiocarcinoma (ICC) is a kind of adenocarcinoma caused by cells in the inner wall of bile ducts in the liver. It has a high mortality rate and a low cure rate. Liver cancer mortality ranks second in China and is the second largest malignant tumor disease in China [1–3]. The pathogenesis of ICC is still unclear, and most scholars believe that the etiology of ICC is mainly related to congenital biliary anomalies, primary sclerosing cholangitis, intrahepatic biliary calculi, parasitic infection, and other factors [4–6]. The main clinical manifestations of ICC include nausea, jaundice, abdominal pain, and night sweats, which seriously threaten the life safety of patients and reduce their quality of life. Due to the occult nature of ICC in its early onset, early detection, early diagnosis, and early treatment are advocated for clinical treatment. Contrast-enhanced ultrasound (CEUS) is a detection method for screening various malignant tumors in clinical practice, but its specificity and sensitivity cannot meet the needs of clinical detection, while enhanced MR scanning can make the development of local lesions in patients more clear. With the continuous improvement of hospital technology, CEUS combined with enhanced MR scanning has been widely used in clinical detection in order to meet the requirements of hospitals for the accuracy of test results [7]. In order to further explore the clinical application effect of CEUS combined with enhanced MR scanning in ICC, 90 cases of patients with ICC admitted to our hospital from June 2017 to June 2018 were selected as the research objects, and the summary report is as follows.

## 2. Materials and Methods

### 2.1. General Information

A total of 90 patients with ICC admitted to Ganyu District People's Hospital of Lianyungang City from June 2017 to June 2018 were selected as the study subjects and randomly divided into control group and experimental group, with 45 cases in each group.

### 2.2. Inclusion Criteria

- Patients with Child-Pugh grade A and B liver function were included [8]
- Complete clinical data
- The study was approved by the Ethics Committee of Ganyu District People's Hospital, and the patients and their families knew the purpose and procedure of the study and signed the informed consent

### 2.3. Exclusion Criteria

- Patients complicated with malignant tumor
- Patients with mental and other cognitive disorders
- Patients with scanning contraindications

### 2.4. Methods

CEUS (Samsung Madison Co., Ltd.; Approval no. 20192062077, Model no. WS80 A) was performed on patients in the control group with a convex array probe frequency between 2.0 MHz and 10.0 MHz. The patients' liver, spleen, kidney, pancreas, and gallbladder were routinely examined by two-dimensional ultrasound to determine the location of tumor lesions. Bile duct dilatation and liver shape and size were observed and recorded. The interference of fluid and lower abdomen gas was reduced by drinking water method and fat meal method. After the detection, the patients were subjected to selective superimposed local amplification of second harmonic imaging with contrast agent sulfur hexafluoride microbubbles (SonoVue, Bracco Suisse SA Shanghai Xinyi Pharmaceutical Co., LTD., Approval no. J20180005, Specification: 59 mg).

The experimental group was detected by CEUS combined with enhanced MR scanning. The detection method of CEUS was the same as that of the control group. The specific detection method of enhanced MR scanning was as follows: the patients were forbidden to drink water 6 hours and eat 12 hours before examination. A superconducting MR scanner (ROYAL PHILIPS; Approval no. 2015 no.3282757; Model: Ingenia II 3.0 T) was used for detection. Routine T1WI and fat-suppressed T2WI images were performed to obtain sagittal, coronal, and cross-sectional images. The scanning area was from the top of the septum to the pelvic cavity. Gadolinium injection (Bayer Schering Pharma AG; Approval no. J20080063) was administered intravenously. The injection dose was 0.2 mL/kg (or 0.1 mmol/kg) per body weight, and the maximum dosage was 0.4 mL/kg per body weight. The patients were scanned for the arterial phase 20 seconds after injection, the portal vein phase 50 seconds after injection, and the delayed phase 4 minutes after injection.

### 2.5. Observed Indicator

The detection results of patients in the two groups were compared, including the detection rate of lesions, localization accuracy, qualitative accuracy, and diagnostic coincidence rate.

Benign and malignant indicators of the two groups were compared, including lesion length, tube wall thickness, and enhancement ratio of triple-phase multislice CT scan of the third stage.

### 2.6. Statistical Analysis

In this study, SPSS20.0 was selected as the data processing Software, and GraphPad Prism 7 was used to graph the data. *χ*^2^ test, *t*-test, and normality test were adopted. When *p* < 0.05, the difference was statistically significant.

## 3. Results

### 3.1. Comparison of General Information

There were no significant differences in gender, age, BMI, average course of disease, smoking, drinking, and residence between the two groups (*p* > 0.05, Table 1).

### 3.2. Comparison of Detection Results between the Two Groups

The rate of lesion detection, accuracy of localization, qualitative accuracy, and diagnostic coincidence rate of the experimental group were significantly better than those of the control group (*p* < 0.05, Table 2).

### 3.3. The Length of Lesions Was Compared between the Two Groups

The length of lesions in the experimental group (9.37 ± 3.12 mm) was significantly smaller than that in the control group (14.88 ± 4.23 mm) (*p* < 0.001, Figure 1).

### 3.4. Comparison of Tube Wall Thickness between the Two Groups

The thickness of tube wall in the experimental group (2.33 ± 0.57 mm) was significantly lower than that in the control group (4.86 ± 0.85 mm) (*p* < 0.001, Figure 2).

### 3.5. The Enhancement Ratio of Triple-Phase Multislice CT Scan Was Compared between the Two Groups

The enhancement ratio of triple-phase multislice CT scan in the experimental group was 24.44%, which was significantly lower than the control group (44.44%, *p* < 0.05, Figure 3).

A, in the experimental group, 11 (24.44%) and 34 (75.56%) patients were with triple-phase high enhancement, while 34 (75.56%) patients were without enhancement.

B, in the control group, 20 patients (44.44%) were with triple-phase high enhancement, and 25 patients (55.56%) were without enhancement.

### 3.6. CEUS Image of ICC Patients

The CEUS images of ICC patients in the experimental group are shown in Figure 4.

### 3.7. MR Images of ICC Patients

MR images of ICC patients in the experimental group are shown in Figure 5.

## 4. Discussion

ICC is occult in the early stage, and the clinical manifestations lack specificity, so it is difficult for doctors to determine the symptoms of patients during detection, and misdiagnosis and missed diagnosis often occur [9, 10]. Delayed diagnosis often leads to the loss of the best treatment opportunity, which seriously threatens the life safety of patients and reduces the quality of life of patients. In recent years, CEUS has been widely used in clinical detection. However, the sensitivity and accuracy of CEUS images are still uncertain due to the few studies on ICC. According to the image analysis, most scholars found that although there were no obvious characteristics in the sonogram of ICC. However, there were visible invasive growth masses, accompanied by varying degrees of hilar lymph node enlargement, bile duct dilation, and intrahepatic bile duct stones [11, 12]. Therefore, most hospitals use enhanced MR scanning, which has relatively mature diagnostic technology with high image contrast and strong capability of qualitative diagnosis of ICC. The diagnosis of ICC by enhanced MR scanning can be differentiated by intrahepatic diseases such as hepatocellular carcinoma, bacterial liver abscess, and enhanced characteristics.

Although CEUS detection provided a basis for doctors' diagnosis, but the expected effect was not achieved [13], the difference of CEUS combined with enhanced MR scanning can provide scientific data and information for ICC, and the detection results are more accurate [14, 15]. The results of this study showed that the lesion length and tube wall thickness of the experimental group were significantly better than those of the control group, which were similar to the results of [16]. Compared with single detection, CEUS combined with enhanced MR scanning detection results are more accurate. In addition, the enhancement ratio of triple-phase multislice CT scan in the experimental group was significantly lower than that in the control group, which was similar to the results of [17]. Moreover, the study has confirmed that the detection rate of CEUS combined with enhanced MR scanning was higher. The detection rate of lesions, localization accuracy, qualitative accuracy, and diagnostic coincidence rate in the experimental group are significantly better than those in the control group, which was similar to the results of [18]. Our results indicated that CEUS combined with enhanced MR scanning was more accurate and comprehensive in the diagnosis and differentiation of ICC. However, there are still some shortcomings and deficiencies in this study. For example, the sample size is too small, which may lead to inaccurate results. In addition, the correlation between CEUS combined with enhanced MR scanning and ICC staging remains to be verified in further clinical trials.

## 5. Conclusion

In conclusion, CEUS combined with enhanced MR scanning has high sensitivity and specificity and can provide scientific detection data for doctors. Compared with the single detection method, CEUS combined with enhanced MR scanning can effectively improve the accuracy of ICC detection.

## Figures and Tables

**Figure 1:** The length of lesions was compared between the two groups. ^*∗∗∗*^*p* < 0.001.

**Figure 2:** Comparison of tube wall thickness between the two groups. ^*∗∗∗*^*p* < 0.001.

**Figure 3:** Comparison of enhancement ratio of triple-phase multislice CT between the two groups.

**Figure 4:** CEUS of ICC patients. (a) High enhancement in arterial phase (arrow direction). (b) The lesions showed low echo under two-dimensional ultrasound (arrow direction).

**Figure 5:** MR image of ICC patients. (a) MR enhanced portal vein phase and other enhancement. (b) MR enhancement delay period high enhancement.

**Table 1:** Comparison of general data between the two groups.

	Experimental group (*n* = 45)	Control group (*n* = 45)	*χ* ^2^ or t	*p*
*Gender*			0.185	0.667
Male	28 (62.22)	26 (57.78)		
Female	17 (37.78)	19 (42.22)		
Age (years)	54.33 ± 3.6	55.17 ± 3.3	1.153	0.251
BMI (kg/m^2^)	24.56 ± 1.76	25.12 ± 1.53	1.610	0.110
Average course (months)	6.21 ± 3.25	6.19 ± 3.33	0.028	0.977
*Smoking*			0.045	0.833
Yes	24 (53.33)	23 (51.11)		
No	21 (46.67)	22 (48.89)		
*Drinking*			0.182	0.670
Yes	27 (60.00)	25 (55.56)		
No	18 (40.00)	20 (44.44)		
*Living area*			0.442	0.506
City	31 (68.89)	28 (62.22)		
Village	14 (31.11)	17 (37.78)		

**Table 2:** Comparison of detection results between the two groups [*n* (%)].

	n	The rate of lesion detection	Accuracy of location	Qualitative accuracy	Diagnose accordance rate
Experimental group	45	100% (45/45)	100% (45/45)	97.78% (44/45)	97.78% (44/45)
Control group	45	82.22% (37/45)	80.00% (36/45)	75.56% (34/45)	77.78% (35/45)
*χ* ^2^		8.780	10.000	9.615	8.389
*p* value		＜0.05	＜0.05	＜0.05	＜0.05

## Data Availability

The datasets used and/or analyzed during the current study are available from the corresponding author on reasonable request.
